The article "The Status Quo of Criminal Responsibility for Aflatoxin Pollution in China: From the Perspective of Judgment Analysis" was retracted in 2023. Reasons: unreliable results or conclusions; concerns about the data; concerns about the peer review; concerns about the citations.

# The Status Quo of Criminal Responsibility for Aflatoxin Pollution in China: From the Perspective of Judgment Analysis

**DOI:** 10.1155/2022/8212370

**Published:** 2022-08-10

**Authors:** Peipei He, Qiaoling Yang, Chenjing Wang, Ying Huang

**Affiliations:** School of Law, Fuzhou University, Fuzhou 350108, China

## Abstract

With the development of the economy, the food safety problems caused by aflatoxin have become increasingly prominent. With regard to the control of aflatoxin pollution, the Chinese government has promulgated a series of legal documents on food safety related to aflatoxin pollution, such as the formulation of industry standards for allowable limits of aflatoxin and various penalties for violators. Although these measures have achieved good results to some extent, there are still many legal problems. This study reviews the current situation of aflatoxin pollution control in food in China. The court judgment documents related to aflatoxin pollution from January 1st 2014 to January 1st 2020 are investigated to analyze the accountability status of aflatoxin pollution treatment in China. Furthermore, this study mainly cross verified the above problems by means of the literature survey and an organization interview and proposed solutions on the basis of in-depth analysis of their causes. Finally, some suggestions are put forward to solve the problem of aflatoxin pollution accountability in China.

## 1. Introduction

Aflatoxin (AFS) is a kind of toxic secondary metabolite produced by *Aspergillus flavus*, *Aspergillus parasiticus,* and other fungi. So far, more than 20 types of AFS have been identified, including AFB1 and afb2 and AFG1 and afg2, as shown in Figure 1 and 2. Aflatoxin was first discovered in the 1960s. Subsequently, more and more studies have shown that these toxins pose a serious threat to human and animal health. Aflatoxin poisoning caused by eating moldy food has been reported at home and abroad [1]. For example, in 1960, 100,000 turkeys died suddenly in Britain within a few months, which was proved to be caused by *Aspergillus flavus*. In 1974, in Western India, 397 people suffered from acute hepatitis and 106 died from eating corn contaminated with *Aspergillus flavus*. At the beginning of 2004, 317 people in eastern Kenya suffered from liver failure and 125 died from eating corn contaminated by *Aspergillus flavus*. So far, aflatoxin contamination of food has become a worldwide safety problem, especially in developing countries such as Uganda and India [2]. Many countries are working together to ensure that this problem is solved. The latest statistical data released by the Food and Agriculture Organization (FAO) of the United Nations shows that the annual mycotoxin pollution rate of global agricultural products has been rising, which may reach 25% in some cases [3]. Especially, wheat, rice, sorghum, peanuts, and soybeans are more vulnerable to pollution [4]. So far, aflatoxin has existed in the world for more than half a century. Countries have also established allowable limit standards for most mycotoxins, including aflatoxin in food, to ensure the safety of humans and animals.

The article "The Status Quo of Criminal Responsibility for Aflatoxin Pollution in China: From the Perspective of Judgment Analysis" was retracted in 2023. Reasons: unreliable results or conclusions; concerns about the data; concerns about the peer review; concerns about the citations.

The remainder of this paper is organized as follows.  Section 2 discusses the related work, followed by the processing of court documents and data in Section 3. The results and analysis are discussed in Section 4.  Section 5 concludes the paper with a summary.

## 2. Related Work

There are currently a large number of published studies in various countries focusing on the harm caused by aflatoxins to humans and animals. The results showed the toxicity of aflatoxin is equivalent to 10 times that of potassium cyanide, 68 times that of arsenic, and 100 times that of dichlorvos, which is very harmful to the liver and kidneys of humans and animals.

Human ingestion of food contaminated with this toxin can induce primary liver cancer, stomach cancer, and lung cancer. Although all these studies outline the major concerns of aflatoxins worldwide and subsequent countermeasures to limit their contamination levels, there is no consensus on how to prevent and deal with this problem. Some scholars, such as Lauer et al. [5], Ezekiel et al. [6], and Leonmartinez et al. [7], have explored the harmful effects of aflatoxins on animals and humans, focusing on physical and chemical characteristics. Besides, some studies, such as Assaf et al. [8], Nazarizadeh et al. [9], and Wacoo et al. [10] expressed concerns about developing strategies to biologically prevent and inhibit the contamination and growth of aflatoxins in food. In the field of food science, Bandyopadhyay et al. [11] and Ezekiel et al. [12] explored the reduction of the effect of aflatoxin intake in humans once it is ingested. Most recent studies have been conducted to explore the effect of the external environment on changes in aflatoxin content in foods [13–15]. In addition, some research work has made great progress in the degree and severity of aflatoxin contamination to food and common detection methods in various fields [16–18].

It is worth noting that all the above-mentioned studies are in the field of natural sciences. Although all these studies have played a valuable role in helping to understand, prevent, and control the levels of harm caused by aflatoxins, some of the social problems caused by aflatoxins cannot be solved solely by scientific methods. It is believed that this article will be of great help to both policymakers and researchers in academia seeking to legally improve the control of aflatoxins in China and establish a strong reference for other countries around the world. It will also help the food safety supervision and management agencies to improve their administrative work in accordance with the law while also providing some useful insights that would help to improve the country's relevant legislation in the field of food safety.

The article "The Status Quo of Criminal Responsibility for Aflatoxin Pollution in China: From the Perspective of Judgment Analysis" was retracted in 2023. Reasons: unreliable results or conclusions; concerns about the data; concerns about the peer review; concerns about the citations.

## 3. Processing of Court Documents and Data

To draw reasonable conclusions and offer practical solutions, all kinds of judgments (civil judgments, criminal judgments, and administrative judgments) and documents relevant to cases involving aflatoxin contamination in China were collected and analyzed to determine the currently existing problems. In addition, in-depth interviews were organized and the emphasis was placed on the core issues to be able to provide reasonable solutions.

### 3.1. Selection of Court Documents/Interviewees

In this study, several court verdicts related to aflatoxin contamination and control in China were collected and analyzed. Court verdict refers to the legally effective judicial document provided by the People's Court after the court has exercised its judicial power on behalf of the state, which truthfully records the process and the results of the trial and clearly reflects every party' (e.g., judges, prosecutors, administrative officers, defendants, and victims) understanding of the case and the attitudes during the law enforcement proceedings [19].

Currently, the China Judgments Online contains the largest number of court verdicts/documents in China. Up to October 31st 2018, about 55.13 million court verdicts had been uploaded on the website and the total number of visits had reached 20.014 billion [20]. By using the term “aflatoxins contamination” as the keyword, the search results of full-text on this website are about 371 in total, which collects all related court verdicts from January 1st 2014 to January 1st 2020. Subsequently, in-depth interviews were organized with people with first-hand information, which further helped us to gain additional insights into certain social phenomena, discuss their forming process, and envisage relevant solutions for identical social problems [21].

In order to summarize the valuable reasons and suggestions, both face-to-face and telephone interviews were carried out with 41 highly experienced administrative officers, court judges, prosecutors, and scholars who have personally handled cases related to aflatoxin contamination in the country.

### 3.2. Processing of Court Documents and Data

To better reflect the current status and problems of aflatoxin contamination control in China, a qualitative and quantitative analysis of the case materials was conducted. First, a statistical analysis of the annual number and distribution of cases in the country was conducted to gain insight into the current intensity and frequency of accountability for aflatoxin contamination in the country. Second, the details of the different cases were organized into different categories based on their level of similarity and summarized to provide a good grip on the severity of the problem. Third, a statistical analysis of the results of the court verdicts was conducted, and the trials of the cases in various regions were comparatively analyzed. Finally, both the evidence chain and the trial logic of the courts were analyzed.

The article "The Status Quo of Criminal Responsibility for Aflatoxin Pollution in China: From the Perspective of Judgment Analysis" was retracted in 2023. Reasons: unreliable results or conclusions; concerns about the data; concerns about the peer review; concerns about the citations.

Aiming at the interviews' records, the interviewees' responses were analyzed, and then the contents were summarized outlining the different problems reported by the interviewees and their subsequent suggestions for lasting improvement.

## 4. Result, Analysis, and Discussion

### 4.1. Analyzing the Courts Judgments Related to the Control of Aflatoxins

It is clearly evident that the analysis of the judgments rendered by the People's Courts could help us to understand the current status and existing problems of the aflatoxin control system in China. Also, it provides empirical data that can be subsequently applied to solve those problems.

The judgments related to aflatoxin control from January 1st 2014 to January 1st 2020 were collected from the China Judgments Online (https://wenshu.court.gov.cn/). They were all 371 in total, among them, 25 in 2014, 50 in 2015, 67 in 2016, 75 in 2017, 90 in 2018, and 64 in 2019, as shown in Figure 3.

Referring to the distribution of the different types of cases, there were 105 criminal cases, 225 civil cases, and 41 administrative cases. The data illustrating the distribution of case types, as shown in Figure 4.

Owing to the different nature of three types of cases, the research group analyzed the judicial status quo of those different categories of cases separately: (1) analysis of China's aflatoxin contamination-related civil cases; (2) analysis of China's aflatoxin contamination-related criminal cases; (3) analysis of China's aflatoxin contamination-related administrative cases. This will help to reflect the control of aflatoxin pollution from different aspects of the law.

### 4.2. Alignment of the Country's Aflatoxin Limitation Standards with International Standards

The literature indicates that most of the food safety problems in China are usually caused by insufficient and inappropriate food safety standards [22]. To effectively control the aflatoxin contamination in the country, the related limit standards should be improved to be consistent with advanced international standards. Currently, the legal standards for aflatoxins in China contain 4 national standards (GB), as shown in Table 1. According to the Standardization Law of the People's Republic of China, national standards are compulsory, and the other two types are just recommended. In recent years, China has constantly updated these standards.

The article "The Status Quo of Criminal Responsibility for Aflatoxin Pollution in China: From the Perspective of Judgment Analysis" was retracted in 2023. Reasons: unreliable results or conclusions; concerns about the data; concerns about the peer review; concerns about the citations.

### 4.3. Improvement of Relevant Food Safety Legislation in China

The effective control of aflatoxin contamination in the country depends on the systematical and effective food safety legislation. However, China has no unified laws and regulations on aflatoxin pollution control rules. Some specific measures are scattered in different legal documents, for example: Product Quality Law, Food Safety Law, Agriculture Law, Consumer Protection Law, and Civil Code of People's Republic of China. Moreover, many rules have no implementation rules. There is no good correlation between rules, sometimes even contradictory. For example, if someone buys some products containing excessive aflatoxin, according to the provisions of the food safety law, the person can sue the manufacturer or distributor to compensate for their losses, up to ten times the maximum compensation price or three times the resulting losses. However, if the lawsuit is brought according to the Civil Code of People's Republic of China, the compensation claimed by the plaintiff should be strictly based on the real damage. This kind of contradictory stipulations in the same legal system has led to nonunified law enforcement and different judgment procedures. In addition, most of the existing legal stipulations governing the control of aflatoxins in the country in principle are probable, which is also one of the reasons for the problems in judicial practices, such as inconsistent evidence chains and different judgments in the similar case and in some cases very confusing.

### 4.4. Intensification of Administrative Law Enforcement in Food Safety

Effective administrative law enforcement can also play an important key role in the control of aflatoxin contamination of food. However, our study uncovered a lot of problems which are, in our view, the main reasons for some of the aforementioned problems. Firstly, at present, China has several different administrative agencies responsible for supervising or solving all food safety problems. Due to the unclear distribution of responsibilities, there are a lot of abuses of power. In some cases, the agency may waive responsibility. This will make it difficult for institutions to form effective cooperation [23]. Secondly, some of the administrative institutions are inclined to adopt the fine to replace the other kind of punishments because they want to relieve their financial pressure. Some even managed the revenue of fines for income-generating purposes to guarantee the accomplishment of their penalty quota [24]. Thirdly, administrative law enforcement is not consistent in its efforts to enforce the law. The agency tends to only do some random control, leaving a lot of illegal practices unchecked. Moreover, the precaution and prevention mechanisms of food safety issues are still lacking.

The article "The Status Quo of Criminal Responsibility for Aflatoxin Pollution in China: From the Perspective of Judgment Analysis" was retracted in 2023. Reasons: unreliable results or conclusions; concerns about the data; concerns about the peer review; concerns about the citations.

### 4.5. Improvement of the Coordination and Cooperation Mechanism between Administrative Law Enforcement and Criminal Investigation Departments

Criminal responsibility is usually regarded as the last defense line for food safety-related issues. The effectiveness of the Justice department in this case largely depends on the accuracy of the evidence chain delivered by the administrative department during the first steps of the investigation [25]. However, our analysis revealed that some of the criminal suspects have been investigated and punished by the administrative agencies, although the administrative officers did not offer the case clues to the criminal investigation department. This clearly hindered the aflatoxin contamination accountability because there was no trace of clues to consider while establishing new measures or handling future similar cases. It has also been found that there were large regional differences in the case transferring practices, which led to a noticeably inconsistent evidence chain during the process of a judicial trial. Therefore, it is urgent to build up some coordination and cooperation mechanisms between the administrative organ (which is known as the “Food and Drug Administrative agency” in China) and the judicial department (which is the “Public Security Bureau” in China) to ensure all suspected aflatoxin-related cases are transferred to the criminal justice department and offenders are brought to justice and given due process.

### 4.6. Intensification of Food Inspection and Testing Systems

It was found that the focus of the work of the Food Safety Administrative Agency in China currently was the investigation into counterfeit and low-quality products such as poisoned rice and counterfeit edible oil [26]. However, people pay little attention to the detection of the internal composition and content of food, which is the key to understanding whether the food contains toxins, especially aflatoxin. Therefore, it is believed that strengthening the inspection and examination of aflatoxins in food should be one of the primary tasks towards effective control of aflatoxin contamination and regulation in foodstuffs.

The article "The Status Quo of Criminal Responsibility for Aflatoxin Pollution in China: From the Perspective of Judgment Analysis" was retracted in 2023. Reasons: unreliable results or conclusions; concerns about the data; concerns about the peer review; concerns about the citations.

### 4.7. Enhancement of Educational Awareness of Food Safety against Aflatoxins

All documents analyzed revealed that most of the offenders had low education levels with a slightly weak law-abiding consciousness. At the same time, a large number of consumers still preferred to buy food directly from farmers, vendors, peddles, and other small operators, which was mainly because of their traditional thinking [27]. Typically, people believe that food from farmers is fresher and does not carry a lot of preservatives or additives. Indeed, this kind of lifestyle is transmitted from generation to generation and cannot be changed in a very short time, which increases the possibility for citizens to consume the aflatoxin contamination products. Therefore, to eliminate this kind of habit and decrease the food safety-related incidents, it is important to conduct extensive and systematic educational activities and popularize people's awareness of food security.

## 5. Conclusions

In this study, the judgment cases reported regarding the contamination of aflatoxins in food in China are analyzed. The analysis results reveal that there are currently a small number of cases related to the control of aflatoxins in China, despite the fact that there are often reported cases of aflatoxins in the country. We also observe that there are significant regional gaps in accountability and limited responsibility as well as weak accountability levels. There are many reasons for these differences, including the disunity of the evidence chain and the difference between the aflatoxin limit standard and the international standard. Furthermore, some suggestions are put forward. First, all relevant food safety legislation should be improved. Second, food safety and administrative law enforcement should be improved. Third, the execution link system should be improved. Finally, the food inspection and testing systems should be strengthened, and food safety education should be promoted to create awareness on aflatoxin contamination and prevention. Aflatoxin contamination is not only a food safety problem in China but also an international food safety problem. It is believed that the results documented in this study will be conducive to promoting the solution of aflatoxin contamination in China and even other countries around the world.

## Figures and Tables

**Figure 1:** Chemical structure of AFB1 and AFB2.

**Figure 2:** Chemical structure of AFG1 and AFG2.

**Figure 3:** Trend of variability in the number of documents/litigations related to the control of aflatoxins in China.

The article "The Status Quo of Criminal Responsibility for Aflatoxin Pollution in China: From the Perspective of Judgment Analysis" was retracted in 2023. Reasons: unreliable results or conclusions; concerns about the data; concerns about the peer review; concerns about the citations.

**Figure 4:** The distribution of the case types related to the control of aflatoxins in China.

**Table 1:** National standard for aflatoxin.

No.	Standard number	Standard name	Release date	Implementation date
1	GB/T 36858–2018	Determination of aflatoxin *B*1 in feed high performance liquid chromatography	2018-09-17	2019-04-01
2	GB/T 30955–2014	Determination of aflatoxin *B*1, *B*2, *G*1 and *G*2 in feed by immunoaffinity column purification high performance liquid chromatography	2014-07-08	2015-01-10
3	GB/T 17480–2008	Determination of aflatoxin *B*1 in feed by enzyme linked immunosorbent assay	2008-11-21	2009-02-01
4	GB/T 18980–2003	Determination of aflatoxin *M*1 in milk and milk powder immunoaffinity chromatography purification high performance liquid chromatography and fluorescence spectrophotometry	2003-02-21	2003-08-01

## Data Availability

The simulation experiment data used to support the findings of this study are available from the corresponding author upon request.
